# Potential Benefits of Jujube (*Zizyphus Lotus* L.) Bioactive Compounds for Nutrition and Health

**DOI:** 10.1155/2016/2867470

**Published:** 2016-12-07

**Authors:** Souleymane Abdoul-Azize

**Affiliations:** Department of Pharmacy, Research Group “Integrated Cellular Renewal and Microenvironment”, MERCI UPRES EA 3829, University of Rouen, 76183 Rouen Cedex, France

## Abstract

*Zizyphus lotus*, belonging to the* Rhamnaceae* family, is a deciduous shrub which generally grows in arid and semiarid regions of the globe. In traditional medicine,* Z. lotus* is used as antidiabetes, sedative, bronchitis, and antidiarrhea by local populations. Recently, several scientific reports for health benefit and nutritional potential of bioactive compounds from this jujube have been reported. This plant is rich in polyphenols, cyclopeptide alkaloids, dammarane saponins, vitamins, minerals, amino acids, and polyunsaturated fatty acids. These identified compounds were supposed to be responsible for most of* Z. lotus* biologically relevant activities including antimicrobial, anti-inflammatory, hypoglycemic, antioxidant, and immunomodulatory effects. The aim of the present review was to give particular emphasis on the most recent findings on biological effects of the major groups of* Zizyphus lotus* components and their medical interest, notably for human nutrition, health benefit, and therapeutic impacts.

## 1. Introduction

*Zizyphus Lotus (Z. Lotus)*, also known as jujube, belongs to the angiosperm* Rhamnaceae* family. This family includes about 135–170 species of Zizyphus [1]. As a tropical and subtropical plant,* Z. Lotus* grows generally in arid and semiarid countries and is widely distributed in China, Iran, Africa, South Korea, and Europe like Cyprus, Spain, Greece, and Sicily [2–4]. In Africa,* Z. Lotus* is widely distributed in Mediterranean region, like Algeria, Morocco, Tunisia, and Libya [5]. This plant is employed in nutrition, health, and cosmetics in several forms, for example, honey, tea, jam, juice, oil, loaf, and cake. In addition, in traditional medicine, both in North Africa and Middle East, several parts of* Z. lotus* are given as antiurinary troubles agents, antidiabetes, skin infections, antifever, antidiarrhea, insomnia agents, sedative, bronchitis, and hypoglycemic activities [6–9]. On the other hand, this plant offers a delicious read fruit (jujube) that was consumed fresh, dried, and processed as food by local populations in substantial amounts [10].

In recent years, several scientific reports have been carried out about the presence of many biologically active molecules from* Z. lotus*, which may have high potential benefit in human nutrition, health, and disease [11, 12]. In herbal medicine, the properties of bioactive compounds from plants depend on the part of the plant concerned (root, leaf stalk, pulp, or fruit) and the type of extract used.* Z lotus* is known for its high content in polyphenols exhibiting antioxidant and antimicrobial, immunomodulatory properties [13, 14]. Importantly, others biologically active molecules, particularly cyclopeptide alkaloids, termed lotusines [15–17], dammarane saponins [12], and various flavonoids [18] have been isolated from this shrub, along with polyunsaturated fatty acids (oleic acid and linoleic acid), high carbohydrate, and fibers which are abundant in seed extracts and endowed with antiulcerogenic and antioxidants effects [11, 19].

This review is devoted to the most recent findings on biological effects of the major compounds isolated from different parts of* Z. lotus* and to the different usages of this plant in human foods, health promoting, and disease prevention.

## 2. General Compound Content of* Z. lotus*

*Z. lotus* fruit contains substantial amounts of glutamic acid, mineral matter, sterols, vitamins, tocopherols, fibers, amino acids, triacylglycerol, fatty acid, carbohydrate, and antioxidant compounds (phenols, flavonoids, etc.) which have been supposed to be responsible for most of its health benefits such as hypoglycemic, gastroprotective, immunomodulatory, and antioxidant properties [14, 21, 22]. In this respect, the fruit of* Z. lotus* is a valuable source of nutrients as well as antioxidant [4, 21, 23, 24], antimicrobial, and antifungal [13, 25], immunosuppressive [14], anti-inflammatory [26], and antiulcerogenic [21, 27] compounds.* Z. lotus* leaves contain different carbohydrates and dammarane saponins notably jujuboside B, three jujubogenin glycosides, and jujubasaponine IV [20].* Z. lotus* seeds are used to prepare* lotus* oil enriched in essential fatty acids, liposoluble antioxidants, and many sterols [11].* Z. lotus* root contains four dammarane saponins, large quantity of polyphenol, essential fatty acids, vitamin C, and several cyclopeptide alkaloids, termed lotusines which have a wide range of pharmacological activities including antioxidant, antiproliferative, and antidiabetic activities [12, 15–18, 22, 24, 28]. The pulp of* Z. lotus* contains a significant amount of carbohydrate, phenols, flavonoids, and tannins, which exhibit high antimicrobial activity [19, 25].

## 3. Classification of Natural Biomolecules of* Z. lotus*

As a source of polyphenols, fatty acids, vitamins, and other natural compounds,* Z. lotus* seems to be a potential candidate for human nutrition, health promoting, and disease preventing. An overview of bioactive compounds for each part of* Z. lotus* is presented thereafter.

### 3.1. Major Compounds including Phenols, Flavonoids, Alkaloids, Saponins, and Other Biomolecules

Plant-derived polyphenols are a family of organic molecules. During the last decade, there has been a growing interest in the role of polyphenols, in several human pathologies. They have been shown to possess cardioprotective [30], anticancer, antiviral, antiallergenic, and antispasmodic properties [31, 32]. Given their chemical structure characterized by the presence of many phenolic groups, polyphenols are also able to scavenge reactive radical species and prevent peroxidative reactions [33]. Numerous studies showed their ability to prevent damage of lipids, proteins, and nucleic acids by reactive oxygen and nitrogen species [34–36] and modulate transcription factors [37, 38] and protein tyrosine kinases activation [39, 40].

All parts of* Z lotus* are rich in polyphenol family members such as flavonoids, phenolic acids, and other natural compounds (Table 1). In the fruit, total phenols are the major compound, amounting from 297 to 4078.2 mg/100 g of dry matter; in addition, flavonoids and tannins are present in moderate quantities, 122 and 33 mg/100 g, respectively [13, 23]. In the leaf, total phenol content is 664 mg/100 g [13], along with flavonoids ranging from 130 to 199 mg/100 g [13, 18], high content of saponins (340 mg/100 g) [18], and large amount of carbohydrates (8720 mg/100 g) [20], and other molecules are found in small quantities under 10 mg/100 g (see Table 1). Interestingly,* Z. lotus* seeds contain a very high amount of several compounds such as fats (29.73 g/100 g), fibers (16.57 g/100 g), and protein (14.22 g/100 g) [19], along with carbohydrates (4720 mg/100 g) and small amounts of polyphenol (14.68 mg/100 g) [11]. In* Z. lotus* root bark, polyphenol content is 2009 mg/100 g [24], along with a high content of saponins 219 mg/100 g, high content of flavonoids (120 mg/100 g) [18], and large amount of proanthocyanidins (156 mg/100 g) [24] compared to other molecules such as cyclopeptide alkaloids, amounting from 1.4 to 23.95 mg/100 g [15–17] (Table 1).* Z. lotus* pulp contains high amounts of soluble sugars (10.55 g/100 g), fibers (4.84 g/100 g), mineral matter (3.2 g/100 g), and protein (1.18 g/100 g) [19], along with tannins (922 mg/100 g) and moderate amounts of polyphenol (325 mg/100 g) [25].

In summary, aerial parts (leaves and fruits) of* Z. lotus* are the most important source of polyphenols and flavonoids (3630–8144 mg/100 g) [26], while the seeds are rich in fats [19]. These variations in* Z. lotus* biomolecules content might be due to the environment, soil type, climate, or age of the plant.

It should be noted that the biological activities of* Z. lotus* are allocated to the different classes of pharmacologically active compounds such as flavonoids, several saponins, and alkaloids (Table 1). It has been reported that* Z. lotus* alkaloids exerted significant antifungal and antibacterial properties [12, 17].* Z. lotus* saponins presented antisweet effects [12]. Currently, seven alkaloids (called lotusines, named from A to G) and nine saponins (seven jujubogenins and two lotogenins) (Figure 1 and Table 1) have been isolated from this plant, and the main chemical compounds including lotusine A, lotusine B, lotusine C, jujuboside A, lotoside I, and 3-O-*α*-L-rhamnopyranosyl-(1-2)-[(4-sulfo)-*β*-Dglucopyranosyl-(1-3)]-*α*-L-arabino-pyranosyl-jujubogenin are presented in Figure 2.

### 3.2. *Z. lotus* Fatty Acid Composition

The analysis of lipid composition showed that* Z. lotus* pulp (Table 1) was rich in palmitic acid (C16:0), oleic acid (C18:1), and linoleic acid (C18:2), amounting to 27.59%, 24.52%, and 36.63% of total fatty acid content, respectively (Table 2) [28]. Linoleic acid is considered as essential fatty acids. Its content in* Z. lotus* pulp (36.87%) is thus close to the amount found in olive oil (1.1%) [41] and argan oil (31.3%) [42] but lower to the percentage found in soybean oil (50.1%) [43] and corn oil (56%) [44] (Table 2).

Numerous studies reported that all parts of* Z. lotus* particularly, seeds, pulp, fruits, leaves, almond, root, and stem, were rich in palmitic, stearic, linoleic, and oleic acid [11, 13, 19, 28]. Oleic acid was the most important fatty acid of* Z. lotus* fruits [13], seeds [11], and almond [19] at 88.12%, 61.93%, and 49.88%, respectively.* In vivo* studies in rabbit LDL model provided evidence that oleic acid is responsible of the potent antioxidant properties attributed to many edible oils rich in this fatty acid [45]. Moreover, it has been reported that oleic acid upregulated the expression of breast cancer resistance protein and thereby modulates intestinal retention of several food toxicants [46].* Z. lotus* almond also presented moderate level of linoleic acid (22.97%). This fatty acid is the precursor of arachidonic acid, which has inhibitory effect of colon cancer [47]. Other fatty acids were also present in this plant like linolenic acid (9.15%) particularly in* Z lotus* leaves. Linolenic acid is the precursor of docosahexaenoic acid, known to have potential benefit for health and for other diseases like cardiovascular diseases.

### 3.3. Triacylglycerol Composition of* Z. lotus* Seed Oil

High-performance liquid chromatography (HPLC) analyses of triacylglycerol (TAG) composition show that* Z lotus* seed oil contains several TAG (Table 3). The glycerol-trioleate was the most compound, amounting to 26.48 g/100 g, along with glycerol-palmitate-dioleate with 18.78 g/100 g [11] (Table 3).

It has been shown that many types of TG like glycerol-trioleate, glycerol-palmitate-dioleate, glycerol-dioleate-linoleate, and glycerol-palmitate-oleate-linoleate stabilized oil oxidation [56, 57]. Thus,* Z. lotus* seed represents a natural source of oil for food industry.

### 3.4. Vitamins Composition of* Z. lotus*

The pulp of* Z. lotus* is rich in vitamin C in amounts up to 190.65 mg/100 g, followed by* Z. lotus* seeds, leaves, root, and stem, containing 170.84, 63.40, 47.20, and 24.65 mg/100 g, respectively (Table 4).* Z. lotus* leaves content is high in vitamin E with 155.71 mg/100 g [28], while* Z. lotus*'s seeds are enriched in *β*-tocopherols with 130.47 mg/100 g [11]. A little amount of carotenoids (1.47 mg/100) was found only in* Z. lotus* fruits. Vitamins B1 and B2 were present in* Z. lotus* seeds with 0.03 and 0.08 mg/100 g. Several parts of* Z. lotus* are rich in vitamin A, ranging from 3.8 to 71.63 mg/100 g. Collectively, these data provide evidence that* Z. lotus* might be considered as a source of many vitamins for human food.

### 3.5. Sterols Composition of* Z. lotus*

Plant-derived sterols have been reported to decrease LDL cholesterol level in blood [58]. The quality of vegetable oil is correlated with its sterol contents. The sterol analysis of* Z. lotus* seed oil showed that seven compounds have been identified [11]. Δ^7^-Campesterol was the major compound with 147.82 mg/100 g (51.86% of total sterol), along with *β*-sitosterol and campesterol with 82.10 and 31.89 mg/100 g, respectively (Table 5). Other sterols notably stigmasterol, Δ^5^-avenasterol, Δ^5^, 24-stigmatadienol, and cholesterol are present in small quantities. Total sterols content in* Z. lotus* seed oil was 285.03 mg/100 g. Compared to other vegetable oils, this content is better than Z. jujuba oil (18.56 mg/100 g) [10] and virgin oil (150 mg/100 g) [59] but lower than those measured in Z. zizyphus (291.82 mg/100 g) [54] and soy oil (350 mg/100 g) [60]. It is important to indicate that there is no available data on the sterol content in the other parts of* Z. lotus*; this issue remains to be determined.

### 3.6. Mineral Composition of* Z. lotus*

The mineral analysis of* Z. lotus* fruit showed that calcium, magnesium, and potassium were the predominance compounds with 490.84, 397.91, and 134.99 mg/100 g, respectively, [55] (Table 6). Similar amounts for magnesium and calcium were found in* Z. lotus* pulp [19], while higher contents of these three minerals are present in* Z. lotus* seeds, with amounts ranging from 92.41 to 1349.06 mg/100 g [11, 19].

### 3.7. Amino Acids Composition of* Z. lotus*

Amino acids composition of* Z. lotus* seeds shows that threonine is the major amino acid in this part with 26.73% of total amino acid content, followed by glutamic acid (17.28%), leucine (13.11%), arginine (9.47%), aspartic acid (7.76%), and alanine (4.56%) (Table 7). In* Z. lotus* seed, total proteins represent 14.22% higher than* Z. lotus* pulp with 1.18% [19]. But nowadays, amino composition of* Z. lotus* pulp remains to be elucidated.

## 4. Traditional Uses of* Z. lotus* in Medicine, Nutrition, Health, and Disease

### 4.1. *Z. lotus* in Ancestral Medicine

Several parts of* Z. lotus* have been used in traditional medicine for the treatment of bronchitis, diarrhea, and abscess [61]. In addition, the powder of dried leaves and fruit mixed with water or milk is used for the treatment of boils [62] and the root bark for the treatment of diabetes [16]. The juice from* Z. lotus* root would be efficient in the treatment of eye leucomas [63]. The fruits and the leaves of* Z. lotus* are used as emollient [61] and in the treatment of diarrhea and intestinal diseases [63].

### 4.2. Z. lotus in Nutrition

*Z. lotus* fruits would still be consumed by local population in North Africa. The fruits are dried and processed into flour to make pancakes with very pleasant flavor [64]. The nutritional virtue of* Z. lotus* is mainly based on its composition rich in vitamin E, vitamin C, fibers, fatty acids, amino acids, calcium, magnesium, and considerable amounts of sugars as mentioned above. The vegetable oils are widely consumed in our diet. They contribute to foods flavor, taste, and texture. Consistent with this, it has been reported that* Z. lotus* oil is of high quality, because of its content in unsaturated fatty acids and other bioactive compounds [11].

### 4.3. *Z. lotus* in Health and Disease

Traditional uses of* Z. lotus* have reported several benefits of this plant and its bioactive compounds. Meantime, there has been a growing scientific data to support these beneficial properties of* Z. lotus* through several experimental models devoted to the assessment of* Z. lotus* natural molecules to cure numerous diseases. This plant is rich in polyphenols, flavonoids, tannins, alkaloids, and saponins which have several healthy properties like antidiabetic, hypoglycemic, and gastroprotective actions [21, 22]. As mentioned above, lotusine B, lotusine C, jujuboside A, and jujuboside C are the main active constituents of* Z. lotus* root bark (Table 1) and might exert antibacterial and antifungal activity [65, 66].

## 5. Pharmacological and Biological Activities of* Z. lotus* Compounds

Therapeutic benefits of* Z. lotus* compounds or extracts have been highlighted by several experimental models (cell and animal) through* in vivo* and* in vitro* studies.

### 5.1. Antioxidant and Anti-Inflammatory

Several studies report that the extracts of* Z. lotus* exhibit anti-inflammatory and antioxidant properties. As shown in Table 1,* Z. lotus* is rich in many antioxidant compounds such as phenolic acids, flavonoids, alkaloids, and saponins. These components have been shown to prevent oxidative stress and inflammation by reducing reactive oxygen species (ROS) [69]. Interestingly, numerous* in vitro* studies have demonstrated the capacity of the different parts of* Z. lotus* for scavenging free radicals, for instance, in lipid peroxidation, resulting in cell damage prevention [4, 13, 21, 23, 24, 26]. Moreover, in diabetic rats, the aqueous extract of* Z. lotus* roots and leaves strongly increases the rate of haemolysis and glutathione reductase and decreases catalase activity, glutathione peroxidase, and the status of antioxidant, suggesting that this plant corrected diabetes-induced antioxidant status [22]. Besides, the involvement of glutathione in protein and DNA synthesis, cellular detoxification, and inflammation has been reported [70]. For this reason,* Z. lotus* extract might have potential benefit for cellular protection.* In vitro* data on human T cells suggest that* Z. lotus* fruits have higher antioxidant activities compared to other parts of this plant, followed by leaves, root, and stem [28]. Furthermore, the secondary metabolites of* Z. lotus* administrated orally in carrageenan-induced rat paw edema presented anti-inflammatory effects in dose-dependent manner [62] by inhibiting paw edema and the production of nitrite in lipopolysaccharide-activated RAW 264.7 macrophages without cytotoxicity [18]. These studies sustained that* Z. lotus* biomolecules might have beneficial effects for human health, for example, to reduce or prevent inflammation and oxidative damage.

### 5.2. Antimicrobial and Antifungal

*In vitro* studies have elucidated the effects of* Z. lotus* extracts on the growth of several bacteria and fungi species (see Table 8). They demonstrated that the extracts of* Z. lotus* fruits under etheric and methanolic solvents presented the most bactericidal effects to induce growth inhibition [13, 25]. These antimicrobial activities of* Z. lotus* fruits seem to be mediated by phenolic compounds content in this part of* Z. lotus* as shown elsewhere [71]. Altogether, these reports provided evidence that* Z. lotus* with antibacterial effects might be considered as source of natural biomolecules for producing synthetic bactericides and fungicides.

### 5.3. Antidiabetic and Hypoglycemic

In a Wistar rat model of streptozotocin-induced hyperglycemia [72], hypoglycemic effects of* Z. lotus* indicate that the aqueous extracts of roots presented the most efficient activities compared to* Z. lotus* leaves [22]. This beneficial effect might be correlated with the high quantities of vitamin A observed in leaves and roots of* Z. lotus*. Indeed, it has been reported that insulin sensitivity was improved by vitamin A through activation of insulin receptor and protein tyrosine phosphatase 1B [73]. Moreover, lower amounts of vitamins were observed in diabetic animals compared to control animals [74].

### 5.4. Antiulcerogenic and Gastroprotective

Gastric ulcer is part of gastrointestinal disorder involving inflammation and default of defense mechanism. In many* in vivo* studies, protective effects of aqueous extracts of* Z. lotus* (root bark, leaves, and fruit) administered orally were observed in the lesions of several ulcerogenic induced models in Wistar rat [21, 27]. These reports suggest that the extracts of this plant act as antiulcer agent by reducing gastric acidity and juice secretion.* Helicobacter pylori* is the most common bacterium that can survive in the highly acidic environment of the human stomach involving different digestive diseases such as peptic ulcer, dyspepsia (heartburn, acid indigestion, and nausea) [75, 76], the stomach cancer (adenocarcinoma) [77, 78], and MALT lymphoma [79]. Interestingly, the effect of methanol extract of* Z. lotus* (fruits) has been studied* in vitro* on 22 clinical strains of* Helicobacter pylori*, indicating that this plant has bactericidal effects on these clinical strains [21].

### 5.5. Analgesic and Antispasmodic

In Swiss mice, analgesic effects of aqueous extract of* Z. lotus* root barks were observed in a dose-dependent manner [62]. In acetic acid-induced algesia in mice, analgesic activities were also reported by flavonoid and saponin extracts from* Z. lotus* leaves and root bark* in vivo*, while* in vitro*, this effect is modulated by nitrite production in RAW 264.7 macrophages [18]. In addition,* ex vivo* studies on isolated rat duodenum show that aqueous extract of* Z. lotus* leaves and root bark exerts antispasmodic activities by modulating Ca^2+^ signaling via cholinergic receptors [32].

## 6. *Z. lotus* Phenolic Compounds and Immune System: Mechanisms of Action

Beneficial effects of* Z. lotus* polyphenols on health might be generated by their antioxidant and radical scavenging properties. Interestingly, our previous studies demonstrated that* Z. lotus* polyphenols also modulate human immune cell signaling and exert immunosuppressive effects [14]. As shown in Figure 3, in human T cells,* Z. lotus* polyphenols (ZLP) upregulate thapsigargin- (TG-, inhibitor of Ca^2+^-ATPase) mediated calcium signaling at endoplasmic reticulum level, modulate plasma membrane, and, thus, block the entry of ions, decrease ERK1 and ERK2 activation, diminish cell proliferation and IL-2 expression by arresting S cell cycle, and increase intracellular acidification in dose-dependent manner [14]. ZLP alone do not induce elevation of intracellular calcium concentration, [Ca^2+^]_*i*_, in these cells. Consistent with this,* Z. lotus* might have a potential benefit in human autoimmune diseases.

## 7. Conclusion

Collectively, this review provides updated comprehensive information on* Z. lotus* as a source of several bioactive compounds which hold therapeutic potentialities for human nutrition, health promoting, and disease preventing. As mentioned in Table 8, several scientific papers have clearly reported many biological properties of the different parts of this plant and its constituents through* in vitro* and* in vivo* studies. The potent antioxidant, antimicrobial, and anti-inflammatory effects of* Z. lotus* have been distinctly elucidated. On another side,* Z. lotus* extracts present beneficial effects on metabolic disorders via antidiabetic and hypoglycemic actions.* In vivo* studies showed that* Z. lotus* supplementation might be used to treat gastrointestinal disorders. On the nutritional level, this plant is rich in many nutriments which may be used in various fields such as food, cosmetics, and pharmaceutics.

## 8. Future Perspectives

Although several studies reported the benefit effects of* Z. lotus* in many facets of human nutrition, health, and disease, the exact mechanisms by which* Z. lotus* bioactive compounds exert their biological and pharmacological activities are not yet entirely elucidated.

Therefore, further studies are required to elucidate the effects of* Z. lotus* extracts and active compounds in some unexplored domains such as cancer, metabolic disorders, inflammation, and age-linked diseases as well as their mechanisms of actions.

## Figures and Tables

**Figure 1:** Common structure of jujubogenins (a), lotogenins (b), and lotusines (c) found in* Z. lotus* [12, 15–17, 20].

**Figure 2:** Structure of* Z. lotus* main phytoconstituents. Note: ^*∗*^3-O-*α*-L-rhamnopyranosyl-(1-2)-[(4-sulfo)-*β*-Dglucopyranosyl-(1-3)]-*α*-L-arabinopyranosyl-jujubogenin.

**Figure 3:** Schematic representation of* Z. Lotus* phenolic compounds-induced immune cell signaling. Note: ZLP:* Z. Lotus* polyphenols; TG: Thapsigargin; PHA: phytohemagglutinin (see text for details).

**Table 1:** Distribution and contents of major bioactive compounds including phenols, flavonoids, alkaloids, saponins, and other phytochemicals in the various parts of *Z. lotus*.

*Z. lotus* part	Major component	Content in mg/100 g	Authors
Fruit	Total phenolic acid	297–4078.2	[13, 23]
	Flavonoids	122	
	Tannins	33	

Leaf	Total phenolic	664	[13, 18, 20, 29]
	Flavonoids	130–199	
	Tannins	39	
	Saponins	340	
	Jujuboside B	3	
	3 jujubogenin glycosides	9.33	
	Jujubasaponin IV	2	
	Monosaccharides (glucose, galactose, rhamnose, arabinose, and xylose)	8720	
	Flavonol glycoside	3	
	Rutin	3.66	
	3′,5′-Diglucosylphloretin	3	

Seed	Total carbohydrate	4087	[11, 19]
	Polyphenol	14.68	
	Crud fats	29730	
	Soluble sugars	4100	
	Total fibres	16570	
	Pectins	1350	
	Crud protein	14220	

Root bark	Total flavonoids	120	[12, 15–18, 24]
	Saponins	219	
	Jujuboside A	6.73	
	Jujuboside C	3.96	
	Lotoside I	2.774	
	Lotoside II	1.58	
	Lotusine A	11.56	
	Lotusine B	23.95	
	Lotusine C	23.95	
	Lotusine D	4.2–10	
	Lotusine E	2.9–10	
	Lotusine F	1.4–11.56	
	Lotusine G	1.5	
	Polyphenol	2009	
	Proanthocyanidins	156	

Pulp	Total phenols	325	[19, 25]
	Flavonoids	173	
	Tannins	922	
	Crud fats	790	
	Soluble sugars	10550	
	Total fibres	4840	
	Pectins	2070	
	Crud protein	1180	
	Mineral matter	3200	

**Table 2:** Comparison of the fatty acid composition of *Z. lotus* and other edible oils; compositions are expressed in g/100 g fatty acids.

Fatty acid	C12:0	C14:0	C16:0	C16:1	C18:0	C18:1	C18:2	C18:3	C20:0	C22:0	C22:1	C24:0	references
*Z. lotus* seed oil	—	0.06	9.14	0.13	4.84	61.93	18.31	1.35	0.17	0.73	—	—	[11]
*Z. lotus* seeds	—	0.15	10.8	0.130	5.45	62.79	14.22	1.30	0.1	—	—	0.9	[28]
*Z. lotus* pulp	—	0	27.59	0	11.25	24.52	36.63	0	0	—	—	0	[28]
*Z. lotus* fruits	0.13	0.176	0.716	—	—	88.12	0.48	0.715	0.178	0.116	0.316	—	[13]
*Z. lotus* leaves	—	0	43.41	5.96	22.15	6.30	6.20	9.15	0	—	—	1.54	[28]
*Z. lotus* almond oil	—	0.084	9.025	0.134	7.106	49.88	22.97	0.409	2.367	1.409	—	—	[19]
*Z. lotus* root	—	0	38.76	0	22.00	19.73	13.24	0	0	—	—	3.66	[28]
*Z. lotus* stem	—	0	33.80	0	24.40	21.73	11.10	0	0	—	—	0	[28]
Argan oil	—	0.10	11.7	0.14	4.9	36.6	31.3	0.09	0.33	0.12	—	0.06	[42]
Cactus seed oil	—	—	20.1	1.80	2.72	18.3	53.5	2.58	—	—	—	—	[48]
Olive oil	—	11.5	0.9	1.4	61.9	3.8	1.1	0.23	—	—	—	—	[41]
Prickly pear peel	0.71	1.95	23.1	2.48	2.67	24.1	32.3	9.27	—	0.5	—	0.41	[49]
Cactus cladodes	1.33	1.96	13.87	0.24	3.33	11.16	34.87	33.23	—	—	—	—	[50]
Grape seed oil	—	0.06	8.3	0.1	3	12	67.6	0.3	0.2	0.1	0.02	0.01	[51]
Sunflower oil	—	0.08	7.4	0.09	4.56	25.17	60.15	0.3	—	—	—	0.34	[52]
Soybean oil	—	—	6	0.4	2.2	26.1	50.1	14.5	—	—	—	—	[43]
Corn oil	—	—	13.4	traces	1.5	27.4	56	0.9	0.2	—	—	—	[44]
*R. stricta* seed oil	—	<0.01	5.96	0.18	2.14	27.01	59.03	0.62	0.76	0.50	0.04	0.16	[53]
*Z. jujuba* pulp	4.68	2.91	18.67	8.69	8.43	36.67	10.88	1.63	1.59	0.56	—	—	[10]
Z. zizyphus seed	—	0.14	4.67	0.06	2.64	46.55	40.77	0.36	0.78	0.98	—	—	[54]

**Table 3:** Composition of triacylglycerol (TAG) in *Z. lotus* seed oil; TAG contents are expressed as g/100 g [11].

	Triacylglycerol	Equivalent carbon number	Content in g/100 g
	Fatty acids attached		
Glycerol	Dipalmitic and oleic acids	48	2.87
	Palmitic, oleic, and stearic acids	50	4.69
	Oleic and dilinoleic acids	44	2.20
	Dioleic and linolenic acids	44	6.23
	Palmitic and dilinoleic acids	44	2.65
	Dioleic and linoleic acids + Palmitoleic and oleic acids	46	16.32
	Palmitic, oleic, and linoleic acids	46	9.28
	Dipalmitic and linoleic acids	46	1.32
	Trioleic acids	48	26.48
	Palmitic and dioleic acids	48	18.78
	Stearic and dioleic acids	50	9.12

**Table 4:** Distribution and contents of vitamins in the different parts of *Z. lotus*. Vitamin contents are expressed as mg/100 g.

	Leaves	Seeds	Root	Pulp	Stem	Fruit	Reported by
Vitamin A	13.52	—	6.45	71.63	3.8		[11, 28, 55]
Vitamin B2	—	0.08	—	—	—		
Vitamin C	63.40	31.24–170.84	47.20	190.65	24.65	5.67	
Vitamin B1	—	0.03		—	—	0.039	
Vitamin E	155.71	—	4.7	11.23	4.5		
Carotenoids	—	0.634	—	—	—	1.47	
*α*-Tocopherol	—	—	—	—	—	—	
*β*-Tocopherol	—	130.47	—	—	—	—	
*γ*-Tocopherol	—	—	—	—	—	—	
*δ*-Tocopherol	—	10.60	—	—	—	—	

Total tocopherols		141.07				0.97

**Table 5:** Comparison of sterols composition of *Z. lotus* seed oil and other edible oils. Sterol contents are expressed in mg/100 g.

*Zizyphus species*	*Z. lotus*	*Z. jujuba*	*Z. zizyphus*	References
Cholesterol	1.73	—	0.22	[10, 11, 54]
Campesterol	31.89	2.4	19.24	
*δ* ^7^-Campesterol	147.82	—	—	
Stigmasterol	16.38	4.69	27.32	
*β*-Sitosterol	82.10	10.65	214.32	
*δ* ^5^-Avenasterol	0.57	—	10.41	
*δ* ^7^-Stigmasterol	—	0.82		
Δ^5^, 24-Stigmatadienol	4.45	—	—	
Cycloartenol	—	—	14.15	
Methylene cycloartenol	—	—	3.32	
Citrostadienol	—	—	2.84	
Total sterols	285.03	18.56	291.82	

**Table 6:** Distribution and contents of minerals in the various parts of *Z. lotus*. Mineral contents are expressed as mg/100 g.

Major component	Seeds	Fruit	Pulp	Source
Potassium	92.41–97.92	134.99	134.99	[11, 19, 55]
Calcium	110.58	490.84	—	
Magnesium	153.92–1349.06	397.91	397.91	
Sodium	7.30–17.41	—	11.45	
Iron	1.21	1.33	1.33	
Manganese	7.84	2.17	2.17	
Zinc	1.38	0.44	0.44	
Copper	—	—	—	
Phosphorus	24	—	10.62	

**Table 7:** Comparison of amino acids content in *Z. lotus* seeds and other plants. Amino acid contents are expressed as g/100 g.

Amino acids	*Z. lotus* seed	*Z. jujuba* seed	*O. ficus-indica* seed	Source
Isoleucine	2.85	2.55	6.20	
Leucine	13.11	5.52	9.94	
Lysine	1.55	4.42	6.79	
Glycine	2.67	3.46	5.06	
Phenylalanine	2.65	2.82	5.25	
Threonine	26.73	30.98	1.53	
Valine + Methionine	1.80	4.05	0.7 + 6.02	[11, 67, 68]
Tryptophan	1.36		trace	
Glutamic acid	17.28	10.02	21.68	
Aspartic acid	7.76	6.38		
Tyrosine	2.27	1.59	3.09	
Serine + histidine + Glutamine	4.57	17	11.57	
Alanine	4.56	4.23	4.75	
Arginine	9.47	2.87	6.63	

**Table 8:** Overview of major bioactive effects of *Z. lotus* preparations in different experimental models.

Biological activity	*Z. lotus* part used	*Experimental models*	References
Antioxidant	*Z. lotus* pulp, seed, leaf, root, and stem extracts	*In vitro* studies in jurkat cells	[4, 13, 21–24, 26, 28]
	*Z. lotus* fruits and root extracts	Dpph radical and hydroxyl radical scavenging activities	
	Methanol extracts of Z. lotus leaf and fruit	Dpph (2,2-diphenyl-1-picrylhydrazyl) assay	
	*Z. lotus* extracts from roots and leaves	*In vivo* studies in wistar rats pancreas, liver, and erythrocytes.	
	Hydroalcoholic extracts of *Z. lotus* leaves and fruits	Lipid peroxidation, dpph	
	*Z. lotus* (fruits) methanol extract	Free radical (dpph) scavenging test	

Antimicrobial	Methanol extracts of leaves and fruits	*In vitro* studies in Gram-negative bacteria: Escherichia coli atcc 8739, Salmonella typhimurium nctc 6017, Aeromonas hydrophila ei, and Pseudomonas aeruginosa atcc 27853	[13, 25]
		*In vitro* studies in Gram-positive bacteria: Staphylococcus aureus atcc 29213, Listeria monocytogenes atcc 7644, and Bacillus cereus atcc 1247	
	Etheric, dichlorométhanic, and methanolic extracts of fruit and its active compounds (phenols, flavonoids, and tannins)	*In vitro* studies in bacterial species: Bacillus subtilis, Bacillus cereus, Escherichia coli, Klebsiella pneumoniae, Salmonella typhi, Staphylococcus aureus, Enterococcus faecalis, and Pseudomonas aeruginosa	

Antifungal	Methanol extracts of leaves and fruits	*In vitro* studies: Aspergillus flavus and Aspergillus niger	[13, 25]
	Etheric, dichlorométhanic, methanolic, and difenoconazole extracts of fruit	Fungal species: Penicillium italicum, Fusarium culmorum, Aspergillus ochraceus, and Rhizomucor sp	

Anticandidal	Methanol extracts of leaves and fruits	*In vitro *studies: candida albicans	[13]

immunosuppressive	Polyphenols from *Z. lotus* fruit	*In vitro* studies: human t cells	[14, 28]
	pulp, seed, leaf, root, and stem extracts	*In vitro* studies: jurkat cells	

Anti-inflammatory	Flavonoid and saponin from root bark and leaves of *Z. lotus*	*In vivo* studies in wistar rats and swiss albino mice *In vitro* studies in raw 264.7 macrophages	[18, 26, 62]
	Methanolic extracts of root bark and leaves of *Z. lotus*	*In vivo* studies in mice	
	Hydroalcoholic extracts of *Z. lotus* leaves and fruits	Lipoxygenase assay	

Analgesic	Flavonoid and saponin from root bark and leaves of *Z. lotus*	*In vivo* studies in wistar rats and swiss albino mice	[18, 62]

Antiulcerogenic	Aqueous, methanolic, ethyl acetate, and chloroformic extracts of *Z. lotus* root barks, leaves, and fruit	*In vivo* studies in wistar rats	[21, 27]
	*Z. lotus* (fruits) methanol extract	*In vivo* studies in wistar rats	

Antispasmodic	Aqueous and methanolic extracts of *Z. lotus* leaves and root barks	*Ex vivo* studies on isolated rat duodenum	[32]

Antidiabetic	*Z. lotus* aqueous extracts from roots and leaves	*In vivo* studies in diabetic wistar rats pancreas, liver, and erythrocytes.	[22]

Hypoglycemic	Aqueous extract of leaf and root from *Z. lotus*	*In vivo* studies in wistar rats	[22]

Gastroprotective	*Z. lotus* (fruits) methanol extract	*In vivo* studies in wistar rats	[21]
		*In vitro* studies in 22 clinical strains of helicobacter pylori j99	

## Abbreviations

*Z. Lotus*: * Zizyphus lotus*
ZLP: * Zizyphus lotus* polyphenols
TG: Thapsigargin
PHA: Phytohemagglutinin
[Ca^2+^]_*i*_: Intracellular calcium concentration
IL-2: Interleukin-2
ERK1/2: Extracellular signal-regulated kinase 1/2
ER: Endoplasmic reticulum.
